The article "Let-7a Targeting TNFAPI3 Promotes Vascular Endothelial Cell Apoptosis of Pediatric Patients with Henoch–Schönlein Purpura via NF-κB Signaling Pathway" was published in 2022. Journal: J Healthc Eng.

# Let-7a Targeting TNFAPI3 Promotes Vascular Endothelial Cell Apoptosis of Pediatric Patients with Henoch–Schönlein Purpura via NF-*κ*B Signaling Pathway

**DOI:** 10.1155/2022/3889318

**Published:** 2022-02-26

**Authors:** Mingming Cui, Jilong Liu, Li Geng, Qianqian Li, Leiming Xi

**Affiliations:** ^1^First Clinical College, Shandong University of Traditional Chinese Medicine, No. 4655, Daxue Road, University Science Park, Changqing District, Jinan, Shandong 250355, China; ^2^Department of Pediatrics, Cao County People's Hospital, Qinghe Road East, Fumin Avenue South, Caoxian Development District, Heze, Shandong 274400, China; ^3^Department of Physiotherapy, Jinan City People's Hospital, No. 001, Xuehu Street, Laiwu District, Jinan, Shandong 271199, China; ^4^Department of Second Internal Medicine, Jinan Shizhong People's Hospital, No. 61, Langmaoshan Road, Jinan, Shandong 250002, China; ^5^Department of Pediatrics, Affiliated Hospital of Shandong University of Traditional Chinese Medicine, No. 42, Wenhuaxi Road, Jinan, Shandong 250011, China

## Abstract

**Objective:**

We aimed at exploring the role of let-7a in the pathogenesis of pediatric Henoch–Schönlein purpura (HSP) and its related mechanism.

**Methods:**

Fifty-five pediatric HSP patients and 20 paired healthy controls were included. The expressions of let-7a and TNFAIP3 were detected by RT-qPCR or/and western blot. Vessel fibrinoid necrosis was evaluated in skin tissues by PTAH staining. The serum IgA level was measured by ELISA. Cells were transfected with let-7a inhibitor and/or TNFAIP3 siRNA, accompanied by pretreatment with NF-*κ*B inhibitor PDTC or not. After being cultured in HSP serum, the changes in cell viability, cell apoptosis, apoptosis-related proteins, and NF-*κ*B pathway-related proteins were detected by CCK8, flow cytometry, and western blot.

**Results:**

The let-7a expression level was positively correlated with the serum IgA level and severity degree of vascular fibrinoid necrosis in HSP patients. Let-7a expression was significantly increased, whereas cell viability and TNFAIP3 expression were obviously decreased 48 h after HUVECs were incubated with HSP serum. Let-7a knockdown upregulated the cell viability, whereas it reduced the apoptotic ratio, apoptosis protein expressions (Bax/Bcl2 ratio, cleaved-caspase 3), and NF-*κ*B pathway activation (reflected by reduced P65 nuclear translocation and p-I*κ*B*α* expression) in HUVECs (all *p* < 0.05). The changes induced by let-7a knockdown were obviously reversed by TNFAIP3 siRNA transfection (*p* < 0.05). Besides, PDTC treatment remarkably diminished the anti-apoptosis effect of let-7a knockdown and pro-apoptosis effect of TNFAIP3 siRNA on HUVECs induced by HSP serum.

The article "Let-7a Targeting TNFAPI3 Promotes Vascular Endothelial Cell Apoptosis of Pediatric Patients with Henoch–Schönlein Purpura via NF-κB Signaling Pathway" was published in 2022. Journal: J Healthc Eng.

**Conclusions:**

Let-7a knockdown significantly suppressed vascular endothelial cell apoptosis induced by HSP serum by targeting TNFAPI3 via NF-*κ*B signaling pathway. Our findings provided a potential therapeutic target for the treatment of HSP.

## 1. Introduction

Henoch–Schönlein purpura (HSP), later renamed IgA vasculitis, is a common systemic vascular inflammatory disease mediated by IgA-related immune complex [1]. It is the most common type of vascular inflammation in children, especially for pediatric patients under the age of ten [2]. Vascular endothelial cells were the most affected cells in HSP, and their apoptosis was a significant pathological phenomenon in HSP. Besides, the recurrence rate of HSP is high, up to 94% of all pediatric patients [3]. Currently, the optimal therapy for HSP is controversial; thus, the development of novel effective therapy is urgently needed.

Micro-RNAs (miRNAs), as a group of endogenous noncoding RNAs, modulated the expressions of their target genes by binding to the 3' untranslated regions (UTRs) of genes. Increasing pieces of evidence show that miRNAs play a regulatory role in multiple cellular functions, such as cell proliferation, apoptosis, immunity, and inflammation [4, 5]. Studies have proposed miRNAs as the prognosis, diagnosis, and therapeutic target for diseases [6–8]. Since miR-let-7a was discovered in *Caenorhabditis elegans*, the de-expression of let-7a was found in multiple diseases. A recent study has suggested that let-7a was a target for inducing the apoptosis of lung cancer cells [9]. The serum level of let-7a is suggested as the biomarker for hepatocellular cancer [10]. Besides, Let-7a was found to be downregulated in scleroderma and contributed to the accumulation of type I collagen [11]. Let-7a was upregulated in osteoarthritis, and the downregulation of let-7a exerted function in inhibiting inflammatory injury of chondrocytes [12]. Although let-7a has been reported to exert a protective role in vascular endothelial cells, little is known about the role of let-7a expression in pediatric patients.

Tumor necrosis factor-alpha protein 3 antibodies (TNFAIP3) encoding A20 protein, a ubiquitin editing enzyme, have been found in various types of cells. TNFAIP3 has an anti-inflammatory effect based on ubiquitination function. TNFAIP3 is a key braking mechanism of the immune system. It is reported that the deficiency of TNFAIP3 leads to a severe autoimmune disorder and premature death in mice [13] and silencing of TNFAIP3 showed a harmful effect in vascular cells. Cheng et al. found that the low expression of TNFAIP3 could inhibit the proliferation of mesangial cells in HSP nephritis [14]. In addition, TNFAIP3 plays a negative role in regulating NF-*κ*B signals. The activation of the NF-*κ*B signaling pathway could lead to the apoptosis of vascular endothelial cells [15]. However, the expression and mechanism of let-7a by targeting TNFAIP3 in mediating vascular endothelial cell apoptosis of pediatric HSP have not been strengthened. Therefore, this study aimed at investigating the role of let-7a and underlying molecular mechanism by targeting TNFAIP3 in pediatric HSP patients and provided new therapeutic targets for the treatment of HSP children.

The article "Let-7a Targeting TNFAPI3 Promotes Vascular Endothelial Cell Apoptosis of Pediatric Patients with Henoch–Schönlein Purpura via NF-κB Signaling Pathway" was published in 2022. Journal: J Healthc Eng.

## 2. Methods

### 2.1. Subjects

Fifty-five children (30 males and 25 females, age: 2–10 years) with HSP and 20 healthy subjects (11 males and 9 females, age: 2–11 years) were recruited from the Affiliated Hospital of Shandong University of Traditional Chinese Medicine from March 2015 to November 2018. All the subjects had no history of chronic diseases and malignancy, and the patients' status and information have been tracked for 5 years. The diagnosis of HSP was confirmed according to EULAR/PRINTO/PRES classification criteria. Blood samples and skin biopsy specimens were obtained from treatment-naive patients at diagnosis. Normal skin tissues obtained from the healthy subjects were included as controls. Serum IgA was detected by ELISA kit (Thermo Fisher, Massachusetts, America), and the number of vessel fibrinoid necrosis per mm^2^ in skin samples was evaluated by phosphotungstic acid-hematoxylin (PTAH) staining under light microscopy (Leica, Germany). This study was approved by the ethics committee of our hospital, and all participants or their parents had signed informed consents.

### 2.2. Cell Culture and CCK8 Assay

Human umbilical vein endothelial cells (HUVECs) purchased from the National Institutes for Food and Drug Control (Beijing, China) were incubated in DMEM (Gibco, Carlsbad, USA) containing 10% fetal bovine serum (37°C, 5% CO2). For cell viability analysis, HUVECs were seeded in 96-well plates and cultured with 10% serum samples from HSP patients or healthy controls for 12, 24, 48, and 72 h, respectively. CCK-8 solution 10 *μ*L (Beyotime, Shanghai, China) was added into plates and maintained for 2 h to measure the cell viability at 450 nm.

### 2.3. Real-Time Quantitative RT-PCR (qRT-PCR) Analysis

TRIzol (TaKaRa, Japan) was used to isolate the total RNA from the skin tissue samples and cells. For TNFAIP3 mRNA quantitative analysis, cDNA was synthesized and analyzed by using a One-Step TB Green® PrimeScript™ PLUS RT-PCR Kit (TaKaRa, Japan). *β*-Actin was used as the reference gene. For let-7a quantitative analysis, cDNA was synthesized and analyzed by using Mir-X miRNA qRT-PCR TB Green® Kit (TaKaRa, Japan). The let-7a primer was purchased from Sangon Biotech. The expression levels of TNFAIP3 relative to U6 and let-7a relative to *β*-actin were defined as 2^−△△CT^ values.

The article "Let-7a Targeting TNFAPI3 Promotes Vascular Endothelial Cell Apoptosis of Pediatric Patients with Henoch–Schönlein Purpura via NF-κB Signaling Pathway" was published in 2022. Journal: J Healthc Eng.

### 2.4. miRNA Inhibitor/siRNA Transfection

Let-7a inhibitor, NC inhibitor, TNFAIP3 siRNA, and siRNA-ctrl were transfected to HUVECs by (Lipofectamine 2000) (Invitrogen, California, America). After 24-h transfection, cells were cultured with HSP serum for 48 h. The HUVECs without transfection were used as the controls.

### 2.5. Dual-Luciferase Assay

TNFAIP3 was identified as a target of let-7a by TargetScan (https://www.targetscan.org). To verify the correlation between TNFAIP3 and let-7a, we constructed a luciferase reporter vector, which was introduced with mutated (MUT) or wild-type (WT) 3'UTR of TNFAIP3 targeted by let-7a. The luciferase activity was examined when cells were cotransfected with a let-7a inhibitor.

### 2.6. Flow Cytometry (FCM)

The HUVECs cultured in HSP serum were collected and washed with cold PBS. The cells were incubated with 5 µL of PI and FITC-Annexin V for 15 min in the dark. Finally, the apoptotic ratio of cells was measured by flow cytometer (BD Biosciences, New York, America).

### 2.7. Western Blot

Total protein from HUVECs was isolated with RIPA lysis buffer, and nuclear protein was extracted with nuclei lysis buffer. The protein concentration was determined by the BCA protein kit (Beyotime, Shanghai, China) at 562 nm. Equal amounts of proteins were resolved by SDS-polyacrylamide gels (10%–12% separation gels) and transferred to PVDF membranes (Thermo Fisher, Massachusetts, America). Then, the membranes were blocked with 5% milk for 1 h at room temperature. The membrane was incubated with primary antibodies, such as Bcl2 (1 : 1000, #33–6100, Thermo Fisher, Massachusetts, America), TNFAIP3 (#4625), Cleave-caspase3 (#9664), Bax (#2772), I*κ*B*α* (#4812), p-I*κ*B*α* (#2859), P65 (#8242), P65 in the nucleus (1 : 1000, CST, Boston, America). *β*-Actin (ab8227, 1 : 5000, Abcam, Cambridge, England) was used as an internal control. Then, the membranes were incubated with secondary antibodies (anti-rabbit, #7074, 1 : 1000, CST, Boston, America). The band signals were visualized using the enhanced chemiluminescence kit (Thermo Fisher, Massachusetts, America).

### 2.8. Immunohistochemical Analysis

The paraffin-embedded tissue sections were dewaxed and hydrated by xylene and graded ethanol, respectively. After being blocked with 3% H2O2 and sealed with 10% BSA, the sections were incubated with P65 primary antibody (1 : 400, #8242, CST, Boston, America) overnight and secondary antibody (1 : 1000, #2985, CST, Boston, America) for 1 h. The images were obtained by using a fluorescent microscope.

The article "Let-7a Targeting TNFAPI3 Promotes Vascular Endothelial Cell Apoptosis of Pediatric Patients with Henoch–Schönlein Purpura via NF-κB Signaling Pathway" was published in 2022. Journal: J Healthc Eng.

### 2.9. Statistical Analysis

All the experiments were performed in triplicate. The results were expressed with mean ± standard deviation (SD) and analyzed by GraphPad Prism 7.0, which was one of the most popular software for graph plotting. One-way analysis of variance (ANOVA) or Student *t*-test was used for comparison among more than two groups and between two groups, respectively. The correlation between let-7a and IgA was determined using Pearson's correlation test. The difference with *P* < 0.05 was considered significant.

## 3. Results

### 3.1. The Expression of Let-7a and TNFAIP3 in Skin Samples of HSP Patients and Controls

To determine the potential clinical significance of let-7a and TNFAIP3 expression, qRT-PCR was performed on 55 HSP skin tissues and 20 normal controls. The results revealed that compared with controls, the expression of let-7a was significantly higher and TNFAIP3 expression was obviously lower in the HSP group (all *p* < 0.05, Figures 1(a) and 1(b)). There was an inverse relationship between let-7a and TNFAIP3 expression (Figure 1(c)). The serum level of IgA in HSP patients was measured by ELISA. As shown in Table 1, the serum level of IgA was strikingly upregulated in HSP patients (2688.89 ± 432.98 mg/L), compared to healthy controls (1595.98 ± 385.1 mg/L) (*p* < 0.05). The histopathological changes of the skin in HSP patients were observed based on PTAH staining. According to the average number of fibrinoid necrosis vessels (per mm^2^), 10 patients were classified into 0 to <1 grade, 20 in 1 to <5 grade, and 25 presented with ≥5 vessel fibrinoid necroses. Correlation analysis indicated that the high IgA level was positively correlated with the severity of skin vessel necrosis in HSP patients (*p* < 0.001, Table 1). Additionally, the let-7a expression in HSP patients was upregulated with the increased number of vessel fibrinoid necrosis (*p* < 0.01, Figure 1(d)) and was positively correlated with serum IgA level (*p* < 0.05, Figure 1(e)), which was revealed by Pearson's correlation test. Thus, let-7a expression was positively correlated with IgA-mediated vascular endothelial cell injury in HSP patients.

### 3.2. Let-7a Knockdown Suppressed HUVECs Apoptosis Induced by HSP Serum

To investigate the role of let-7a in vascular endothelial injury in vitro, HUVECs were incubated with 10% HSP serum for 12, 24, 48, and 72 h. Cells cultured with 10% serum of non-HSP subjects were served as controls. As illustrated in Figure 2(a), cell viability was declined time-dependently at 12–48 h after HSP serum culture (*p* < 0.05), whereas no significant decline was observed between 48 and 72 h (*p* > 0.05). And the control serum did not affect the cell viability and behaviors. Additionally, the expression of let-7a showed a time-course increase after HSP serum culture with a peak at 48 h (Figure 2(b)). Thus, cells cultured with HSP serum for 48 h were used for further analysis.

The article "Let-7a Targeting TNFAPI3 Promotes Vascular Endothelial Cell Apoptosis of Pediatric Patients with Henoch–Schönlein Purpura via NF-κB Signaling Pathway" was published in 2022. Journal: J Healthc Eng.

In order to evaluate the effect of let-7a on the apoptosis of vascular endothelial cells in HSP, HUVECs were transfected with let-7a inhibitor or NC inhibitor, followed by exposure to HSP serum for 48 h. The efficiency of let-7a inhibitor transfection was validated by qRT-PCR (Figure 2(c)). CCK8 assay showed that cell viability was obviously elevated after let-7a inhibitor transfection (*p* < 0.01, Figure 2(d)). Based on flow cytometry, the rate of apoptotic cells was remarkably declined in the let-7a inhibitor group compared to NC inhibitor and Blank group (all *p* < 0.01, Figure 2(e)). Parallelly, the expression of cleaved-caspase 3 and Bax/Bcl2 ratio in cells was significantly reduced by let-7a knockdown (all *p* < 0.05, Figure 2(f)).

### 3.3. Let-7a Knockdown Inhibited Apoptosis of HUVECs Induced by HSP Serum via Targeting TNFAIP3

Primarily, we detected the expression of TNFAIP3 in HUVECs cultured with healthy control or HSP serum for 12–72 h. TNFAIP expressions at mRNA and protein level were obviously reduced by HSP serum culture, dropped to the minimum level at 48 h, and remained stable thereafter (*p* < 0.05, Figures 3(a) and 3(b)). The target interaction between let-7a and TNFAIP3 was predicted by TargetScan and determined via a dual-luciferase reporter assay. The luciferase activity of HUVECs transfected with WT TNFAIP3-3'UTR containing binding sequences of let-7a was obviously declined by let-7a overexpression, while there was no significant difference in luciferase activity of cells transfected with MUT TNFAIP3-3'UTR sequences (Figure 3(c)).

Next, to investigate whether let-7a knockdown exerted an inhibitive effect on HUVECs apoptosis via TNFAIP3, HUVECs were transfected with let-7a inhibitor and/or TNFAIP3 siRNA and maintained with HSP serum for 48 h. The obvious increase of TNFAIP3 expression was induced by let-7a inhibitor transfection, which was abolished by cotransfection with TNFAIP3 siRNA (*p* < 0.05, Figures 3(d) and 3(e)). TNFAIP3 siRNA remarkably diminished the increased cell viability of HUVECs induced by Let-7a knockdown under HSP serum treatment (*p* < 0.05, Figure 3(f)). Similarly, TNFAIP3 siRNA obviously reversed the inhibitory effect of let-7a knockdown on HUVEC apoptosis under HSP serum treatment reflected by flow cytometry (Figure 3(g)) and western blot (Figure 3(h)).

### 3.4. Let-7a Knockdown Suppressed HSP Serum-Induced HUVECs Apoptosis by Targeting TNFAIP3 through NF-*κ*B Signaling

TNFAIP3 is a potential NF-*κ*B inhibitor that negatively regulated NF-*κ*B signaling pathway [16]. P65 nuclear translocation and IkB protein phosphorylation are the critical steps for NF-*κ*B pathway activation [17]. We firstly detected the p-I*κ*B*α* expression and the P65 translocation by western blot and/or immunohistochemistry after impaired let-7a and/or TNFAIP3 expression. As shown in Figure 4(a), TNFAIP3 siRNA transfection strikingly increased the expressions of p-I*κ*B*α* and P65 in nuclei of HUVECs under HSP serum culture. Let-7a knockdown significantly reduced the expressions of p-I*κ*B*α* and P65 in nuclei, which was overturned by TNFAIP3 siRNA transfection (*p* < 0.05). The consistent trend of nuclear translocation of P65 was observed in immunohistochemical analysis (Figure 4(b)).

The article "Let-7a Targeting TNFAPI3 Promotes Vascular Endothelial Cell Apoptosis of Pediatric Patients with Henoch–Schönlein Purpura via NF-κB Signaling Pathway" was published in 2022. Journal: J Healthc Eng.

Next, HUVECs were pretreatment with NF-*κ*B inhibitor (PDTC, 50 *μ*mol/L) for 48 h before transfection, followed by treatment with HSP serum for 48 h. The results showed that cell viability was obviously elevated by PDTC treatment and further increased by let-7a inhibitor transfection (all *p* < 0.05). PDTC significantly reversed the suppressive effect of TNFAIP3 siRNA on cell viability (*p* < 0.05, Figure 4(c)). The opposite trend for cell apoptosis was observed by flow cytometry and western blot. As illustrated in Figure 4(d), compared with the NC inhibitor group, the cell apoptotic ratio dropped drastically with let-7a inhibitor transfection (*p* < 0.05). PDTC could enhance the antiapoptotic effect of let-7a inhibitor (*p* < 0.05), while the remarkably abrogated proapoptotic function of TNFAIP3 siRNA in HUVECs (*p* < 0.05). Similarly, a remarkable reduction of cleaved-caspase 3 expression and Bax/Bcl2 ratio were observed in the let-7a inhibitor + PDTC group (*p* < 0.05), whereas PDTC significantly abolished the changed expression of apoptosis-related proteins induced by TNFAIP3 silence (*p* < 0.05, Figure 4(e)). Thus, let-7a knockdown increased the viability and reduced apoptosis of HUVECs by targeting TNFAIP3 via NF-*κ*B signals.

## 4. Discussion

HSP is a clinically common autoimmune vasculitis disease in children aged between 7 and 14 years. However, controversy remains regarding the effective treatment for HSP. Recently, it has been reported that the pathogenesis of HSP might be related to vascular endothelial apoptosis induced by immune molecules [18]. Therefore, suppressing vascular endothelial apoptosis may effectively inhibit the initiation and progression of HSP in children. Thus, in this study, we investigated the expression of let-7a, the relationship with vascular endothelial apoptosis, and the mechanism by targeting TNFAIP3.

The article "Let-7a Targeting TNFAPI3 Promotes Vascular Endothelial Cell Apoptosis of Pediatric Patients with Henoch–Schönlein Purpura via NF-κB Signaling Pathway" was published in 2022. Journal: J Healthc Eng.

As described in a recent study, let-7a was highly expressed in affected tissues of patients with IgA vasculitis [19]. However, the clinical significance has not been clarified. Our data showed that the let-7a level was significantly upregulated in skin lesion tissues of pediatric HSP patients, compared with controls, which was consistent with previous findings. Besides, we found that let-7a high expression was positively correlated with serum IgA level and the severity of vascular fibrinoid necrosis. All these indicated that let-7a might be involved in vascular endothelial apoptosis induced by IgA in HSP children.

Despite the antiproliferative and proapoptotic effects of let-7a on tumor cells that have been reported, the effect of let-7a in HSP children remains relatively uncharacterized. Our data indicated that let-7a expression was elevated by HSP serum culture time-dependently and peaked at 48 h in HUVECs. We speculated that the low expression of let-7a showed an inhibitive effect on vascular endothelial apoptosis in HSP children. Thus, to explore the anti-apoptotic effect of let-7a knockdown on vascular endothelial cells in HSP in vitro, we transfected the let-7a inhibitor into HUVECs and exposed it to HSP serum for 48 h. The data revealed that the let-7a inhibitor served to dampen the HUVECs apoptosis responded to HSP children serum, reflected by elevated cell viability, while it declined the cell apoptosis rate, Bax/Bcl2 ratio, and cleaved-caspase 3 expression. These results indicated that the high expression of let-7a played a key role in vascular endothelial apoptosis of HSP.

However, the potential mechanism by which let-7a promoted HUVECs apoptosis induced by HSP serum remained unclear. TNFAIP3 is a ubiquitin editing enzyme that suppressed the activation of the NF-*κ*B pathway. NF-*κ*B is a transcription factor that plays a critical role in endothelial cell activation by regulating cytokines and related genes and is involved in the death and apoptosis of endothelial cells induced by hypoxia [20]. P65 is a key molecular in the NF-*κ*B pathway, and p65 binds with its inhibiting proteins I*κ*B*α* in the cytoplasm in an inactive form. When NF-*κ*B pathway is stimulated, P65 released from I*κ*B*α* translocates to nuclear and contributes to the phosphorylation of I*κ*B*α* [21, 22]. Our study revealed TNFAIP3 was obviously downregulated in skin lesion tissues of pediatric HSP patients and the HUVECs stimulated by HSP serum. It is suggested that the low expression of TNFAIP3 was related to the pathogenesis of HSP in children. Although previous evidences showed that let-7a modulated the expression of TNFAIP3 in other diseases [23], little is known about the correlation between let-7a and TNFAIP3 in endothelial cells of HSP. In this study, TNFAIP3 was determined to be a functional target of let-7a by luciferase assay. The expression of TNFAIP3 was negatively regulated by let-7a. TNFAIP3 expression was strikingly upregulated by let-7a knockdown. HUVEC apoptosis induced by HSP was observed after cotransfection with let-7a inhibitor and TNFAIP3 siRNA. The results suggested that TNFAIP3 silence could abolish the let-7a inhibitor-suppressed cell apoptosis. The inhibitory effect on the vascular endothelial apoptosis induced by let-7a inhibitor was reversed by TNFAIP3 silence reflected by mitigated cell viability and increased apoptotic ratio. In addition, let-7a inhibitor suppressed I*κ*B*α* phosphorylation and P65 translocation, which was reversed by cotransfection with TNFAIP3 siRNA. These observations primarily indicated that let-7a targeted TNFAIP3 to induce HUVECs apoptosis along with continuous activation of NF-*κ*B signaling.

The article "Let-7a Targeting TNFAPI3 Promotes Vascular Endothelial Cell Apoptosis of Pediatric Patients with Henoch–Schönlein Purpura via NF-κB Signaling Pathway" was published in 2022. Journal: J Healthc Eng.

In order to further demonstrate that let-7a exerted a promotive effect on HUVECs apoptosis by targeting TNFAIP3 via NF-*κ*B pathway, we pretreated HUVECs with PDTC (NF-*κ*B inhibitor) before cotransfection of let-7a inhibitor and TNFAIP3 siRNA. The results revealed that let-7a inhibitor exerted a similar effect with PDTC, contributing to reduced cell apoptosis induced by HSP serum by the blockade of NF-*κ*B activation. However, TNFAIP3 siRNA diminished the antiapoptotic effect induced by let-7a inhibitor + PDTC through reducing cell viability and increasing apoptotic ratio. It is confirmed that let-7a elevated NF-*κ*B activation through directly targeting TNFAIP3 3'UTR to promote HUVEC apoptosis.

## 5. Conclusion

In conclusion, the expression of let-7a was pronouncedly accumulated in the skin lesion tissues of pediatric HSP patients. Knockdown of let-7a significantly inhibited HUVECs apoptosis stimulated by HSP serum through inhibiting NF-*κ*B signaling, which was in turn reversed by silencing the target gene TNFAIP3. Let-7a played a proapoptotic effect on vascular endothelial cells through NF-*κ*B signaling by targeting TNFAIP3. Our findings provided a potential therapeutic target, and intervention of let-7a expression may provide a promising approach for HSP treatment in children. We will continuously look for the upstream and downstream effector molecules of let-7a and investigate their roles and effects in future research.

## Figures and Tables

**Figure 1:** The expression of let-7a and TNFAIP3 in HSP patients. The expressions of let-7a (a) and TNFAIP3 (b) in skin tissues were detected by qRT-PCR analysis. Let-7a was significantly elevated in HSP samples, and TNFAIP3 was downregulated in controls. (c) Negative correlation between let-7a and TNFAIP3 expression in skin tissues by Pearson correlation analysis. (d) The expression of let-7a was detected in HSP patients with different degrees of vessel fibrinoid necrosis. Let-7a expression was upregulated with the increased number of fibrinoid necrosis in HSP patients. (e) Positive correlation between let-7a expression and serum IgA level in HSP patients by Pearson correlation analysis. ^*∗∗*^*p* < 0.01, ^*∗∗∗*^*p* < 0.001. Ns, no significant difference.

The article "Let-7a Targeting TNFAPI3 Promotes Vascular Endothelial Cell Apoptosis of Pediatric Patients with Henoch–Schönlein Purpura via NF-κB Signaling Pathway" was published in 2022. Journal: J Healthc Eng.

**Figure 2:** Let-7a affects apoptosis of HSP serum-induced vascular endothelial cell *in vitro*. Cell viability (a) and let-7a expression (b) were detected in HUVECs treated with 10% HSP serum for 12, 24, 48, and 72 (h) ^*∗*^*p* < 0.05, ^*∗∗*^*p* < 0.01, ^*∗∗∗*^*p* < 0.001, compared with control. Ns, no significant difference. HUVECs were transfected with let-7a/NC inhibitor and exposed to HSP serum for 48, and (h) then, transfection efficiency (c), cell viability (d), cell apoptosis rate (e), and apoptosis-related proteins (f) were evaluated. ^*∗*^*p* < 0.05, ^*∗∗*^*p* < 0.01, ^*∗∗∗*^*p* < 0.001. Ns, no significant difference.

**Figure 3:** Let-7a affects vascular endothelial cell apoptosis by targeting TNFAIP 3. The expressions of TNFAIP 3 in mRNA (a) and protein level (b) were detected by qRT-PCR and western blot, respectively. ^*∗*^*p* < 0.05, ^*∗∗*^*p* < 0.01, ^*∗∗∗*^*p* < 0.001, compared with control. Ns, no significant difference. (c) Target interaction between let-7a and TNFAIP3 was determined by dual-luciferase activity. After cells were transfected with let-7a inhibitor or/and TNFAIP3 siRNA, TNFAIP3 expressions in mRNA, (d) and protein level (e) and cell viability (f) were detected. (g) Cell apoptosis was measured by flow cytometry. (h) The apoptosis-related proteins were detected by western blot. ^*∗*^*p* < 0.05, ^*∗∗*^*p* < 0.01, ^*∗∗∗*^*p* < 0.001. Ns, no significant difference.

**Figure 4:** NF-*κ*B pathway was involved with let-7a modulated vascular endothelial cell apoptosis. (a) The expression of NF-*κ*B pathway-related proteins was detected by western blot. (b) p65 nuclear translocation was detected by immunohistochemistry. (c) Cell viability was detected after cells were treated with let-7a inhibitor, or/and TNFAIP3 siRNA or and NF-*κ*B pathway inhibitor PDTC. (d) Cell apoptosis was measured by flow cytometry. (e) The apoptosis-related proteins were detected by western blot. ^*∗*^*p* < 0.05, ^*∗∗*^*p* < 0.01, ^*∗∗∗*^*p* < 0.001. Ns, no significant difference.

**Table 1:** The correlation between serum IgA level and the number of vessels fibrinoid necrosis in HSP patients.

	Grade	Control (*n* = 20)	HSP (*n* = 55)	*P* value
IgA(mg/L)		1595.98 ± 385.1	2688.89 ± 432.98	*p* < 0.001
Average number of fibrinoid necrosis vessels (per mm^2^)	0 to <1	–	10	-
	1 to <5	–	20	
	≥5	–	25	
Correlation coefficient/*P* value	–	–	*r* = 0.564/*p* < 0.001	-

The article "Let-7a Targeting TNFAPI3 Promotes Vascular Endothelial Cell Apoptosis of Pediatric Patients with Henoch–Schönlein Purpura via NF-κB Signaling Pathway" was published in 2022. Journal: J Healthc Eng.

## Data Availability

The analyzed datasets generated during the present study are available from the corresponding author on reasonable request.
